# Analysis of the Relationship between Nutritional Status and Bone Age and Sexual Development in Children and Adolescents

**DOI:** 10.1155/2022/8325756

**Published:** 2022-08-25

**Authors:** Hong Sun, Weiqun Wang, Shouyuan Zhang, Chenglei Lin

**Affiliations:** Department of Pediatrics, Zhejiang Hospital of Integrated Traditional Chinese and Western Medicine, Hangzhou, Zhejiang 310003, China

## Abstract

**Purpose:**

To observe the correlation between nutritional status, bone age, and sexual development in children and adolescents.

**Methods:**

895 children and adolescents who underwent physical examination in the growth and development clinic and height clinic of our hospital from 2019 to 2021 were selected as the research objects. The subjects were divided into emaciation group, normal group, overweight group, and obesity group. The bone age level, bone age assessment, sexual development, and early maturity rate of each group were compared.

**Results:**

The bone age difference (BAD) of the overweight and obesity groups was higher than that of the normal group, and the BAD of the obesity group was higher than that of the emaciation group (*P* < 0.05). Compared with the normal group, the risk of advancement of bone age in the overweight group increased by 2.674 times (male) and 1.908 times (female), the risk of advancement of bone age in the obesity group increased by 6.376 times (male) and 14.687 times (female), the risk of retardation of bone age in the emaciation group increased by 2.150 times (male) and 3.092 times (female). Whether it was male or female, the sexual development of overweight and obese was higher than that of the normal weight group in the same age group. Among female children, the sexual precocious puberty rate of the overweight + obesity group is higher.

**Conclusion:**

The nutritional status of children and adolescents is closely related to their bone age and sexual development.

## 1. Introduction

The nutritional status of children and adolescents is a sensitive index to measure their health level, and improving the nutritional status of children and adolescents is also an important foundation to improve the quality of the population [1]. Lack of nutrition will not only reduce people's immunity but also directly affect their intellectual development, physical development, psychological development, etc. It will also cause children's physical disharmony, lethargy, poor language expression ability, decreased learning ability, and even cause diseases [2]. In recent years, with the improvement of living standards, the detection rates of overweight and obesity among children and adolescents have been increasing year by year worldwide. Obese children and adolescents are often accompanied by lipid metabolism disorders, which are directly related to the occurrence of hypertension, coronary heart disease, and type 2 diabetes [3]. Obesity has become a serious global public health problem. Studies have predicted that by 2030, the prevalence of overweight + obesity among adults, school-aged children, and preschool-aged children will be 65.3%, 31.8%, and 15.6%, respectively, and the number of overweight + obesity patients will reach 789.95 million, 58.92 million, and 18.19 million, respectively [4]. Lack of nutrition and overnutrition have a long-term impact on children and adolescents, which may reduce the level of physical health in adulthood. At the same time, unhealthy nutritional status will also have a certain negative impact on the psychology of children and adolescents, resulting in psychological problems such as inferiority, being unsociable, loneliness, and irritability [5]. Therefore, ensuring proper nutritional intake of the human body is particularly important for the healthy growth of children and adolescents. Body mass index (BMI) is an important index to measure the body shape that is often used to quickly evaluate the nutritional status. BMI is often used clinically in the field of monitoring and screening children's obesity and thinness [6].

Bone age is an index to evaluate the maturity of skeletal development in children and adolescents. Compared with height, weight, chest circumference and other growth, and development-related indicators, bone age can more accurately reflect the level of individual growth and development [7]. In addition, studies have shown that the initiation of sexual development is related to nutritional metabolism, genetics, environment, and other factors [8]. Precocious puberty is an abnormal growth and development, which is characterized by the early appearance of puberty characteristics. It is generally believed that obesity in children and adolescents is closely related to precocious puberty [9]. At present, the nutritional status, growth and development, and sexual characteristics of children and adolescents have attracted widespread attention. Through physical examination of 895 children and adolescents, this study observed the correlation between their nutritional status, bone age, and sexual development.

## 2. Materials and Methods

### 2.1. Research Object

895 children and adolescents who underwent physical examination in the growth and development clinic and height clinic of our hospital from 2019 to 2021 were selected as the research objects. Inclusion criteria were as follows: 4–17 years old; able to cooperate with physical examination; and clinical data are complete. Exclusion criteria were as follows: severe organic diseases; suffering from genetic syndrome; suffering from congenital malformation; skeletal developmental malformation; severe scoliosis; abnormal sexual differentiation; drugs such as growth hormone and sex development inhibitors that affect the research results are being used; and long-term use of corticosteroids, antihypertensive, and lipid-lowering drugs.

### 2.2. Research Methods

① The height and weight of the subjects were measured by standardized measuring tools and methods. In the measurement of height and weight, it is necessary to carry out quality control. Height measurement is accurate to 0.1 cm and weight measurement is accurate to 0.1 kg. Measuring instruments are verified and calibrated before use. The measurement needs to be carried out three times. Calculate the BMI of the subjects. BMI (kg/m^2^) = weight/height^2^.
② The nutritional status of children and adolescents was assessed according to the classification standards recommended by the WHO. Height and weight < M-2SD are defined as emaciation, BMI > P85 as overweight, and BMI > P95 as obesity.
③ Bone age was judged by X-ray film of the left wrist bone. Bone age assessment was performed by Yitu Children bone age assessment software. Bone age difference (BAD) = bone age−age. −1 year old ≤ BAD ≤ +1 year old is defined as normal bone age development, BAD > +1 year old is defined as advancement of bone age, BAD < −1 year old is defined as retardation of bone age.
④ The development level of sexual characteristics is evaluated by uniformly trained clinicians of the same sex as the examinee, including breasts and pubic hair of girls, external genitalia, testicular volume, and pubic hair of boys. The assessment of breast development in girls was performed by visual inspection combined with palpation, the assessment of testicular volume in boys was performed by palpation, and the assessment of pubic hair development was performed by visual inspection. When the size of the testicles on both sides of the boy is inconsistent, the larger side is selected; when the breast development stages of the two sides of the girl are inconsistent, the more mature side is selected. According to the Tanner staging criteria, girls are divided into B1-5 stages according to breast and pubic hair development criteria, and boys are divided into G1-5 stages according to testicular volume and pubic hair development criteria. Reaching the Tanner stage 2 of development marks the start of puberty development. Precocious puberty is defined as the presence of secondary sexual characteristics in boys under the age of 9. Precocious puberty is defined as the presence of secondary sexual characteristics in girls under the age of 8 or menstrual cramps under the age of 10 [10].

### 2.3. Statistical Methods

SPSS 20.0 software was used for analysis. Measurement data were expressed as mean ± standard deviation, *t*-test or was *F*-test was used to analyze the comparison. When the data met the homogeneity of variance normality, the Bonferroni method was further used for multiple comparisons. Count data were expressed as a ratio, *χ*^2^-test was used to analyze the comparison. The odds ratio (OR) value of risk assessment was calculated using 2 *∗* 2 crosstab data. *P* < 0.05 was statistically significant.

## 3. Results

### 3.1. Age Distribution of 895 Children and Adolescents

A total of 895 children and adolescents were included in the study, including 466 males and 429 females. The age distribution is shown in Table 1.

### 3.2. Nutritional Status and Bone Age Level of Children and Adolescents

The average bone age of emaciation, normal, and overweight groups is consistent with the actual age. There was a significant difference in the BAD of children and adolescents under different nutritional status (*P* < 0.05). The BAD of the overweight and obesity group was higher than that of the normal group, and the BAD of the obesity group was higher than that of the emaciation group (*P* < 0.05). See Table 2.

### 3.3. Nutritional Status and Bone Age Assessment of Children and Adolescents

There was a significant difference in the bone age assessment of children and adolescents under different nutritional status (*P* < 0.05). Compared with the normal group, the risk of advancement of bone age in the overweight group increased by 2.674 times (male) and 1.908 times (female). Compared with the normal group, the risk of advancement of bone age in the obesity group increased by 6.376 times (male) and 14.687 times (female). Compared with the normal group, the risk of retardation of bone age in the emaciation group increased by 2.150 times (male) and 3.092 times (female). See Table 3.

### 3.4. Nutritional Status and Sexual Development of Children and Adolescents

Among male children aged 10 to 12 years, the probability of sexual development in the overweight + obesity group was 1.275 times that of the normal group. Among female children aged 6 to 8 years, the probability of sexual development in the overweight + obesity group was 2.156 times that of the normal group. Among female children aged 8 to 10 years, the probability of sexual development in the overweight + obesity group was 1.114 times that of the normal group. Among female children aged 10 to 12 years, the probability of sexual development in the overweight + obesity group was 1.027 times that of the normal group. See Table 4.

### 3.5. Relationship between Nutritional Status and Early Maturity of Children and Adolescents

No early maturity was found in male children and adolescents. Among female children, the sexual precocious puberty rates of the emaciation, normal, overweight, and obesity groups were 0.00% (0/4), 6.34% (21/331), 15.38% (10/65), and 13.79% (4/29), respectively. See Figure 1.

## 4. Discussion

The growth and development of the human body is a long-term continuous process with a certain law of change and is comprehensively influenced by environmental factors, genetic factors, nutritional status, and other aspects [11]. Nutritional status is one of the important bases for evaluating the physique and health of children and adolescents. Poor nutrition status not only affects people's physical health and increases the risk of diseases but also has certain adverse effects on their normal psychological development [12, 13].

Studies have shown that bone age is not exactly equal to actual age, and bone age can better reflect the overall development degree of individuals [14]. Advanced bone age can lead to early closure of epiphysis in children, which affects the final height, while backward bone age is associated with short stature, delayed sexual development, and other developmental problems [15]. Nutritional status is very important for the growth and development of children's and adolescents' bones. Artioli et al. believed that the average bone age of overweight children is basically consistent with their age, but the bone age of obese children is earlier [16]. In this study, the BAD of the overweight and obesity groups was higher than that of the normal group, and the BAD of the obesity group was higher than that of the emaciation group. It is suggested that overweight and obesity may have a great influence on the bone age of children and adolescents. At the same time, we found that, compared with the normal group, the risk of advance of bone age in the overweight group increased by 2.674 times (male) and 1.908 times (female); the risk of advance of bone age in the obesity group increased by 6.376 times (male) and 14.687 times (female); and the risk of retardation of bone age in the emaciation group increased by 2.150 times (male) and 3.092 times (female). This shows that the rate of bone age retardation in emaciated children is greater than the rate of bone age advancement, and the rate of bone age advancement in overweight and obese children is greater than the rate of bone age retardation. The possible reasons are as follows: ① studies have found that obese children have high levels of leptin. Leptin is a peptide hormone secreted by adipocytes, which has an interaction relationship with other hormones in the body, such as insulin, thyroid hormone, sex hormone, and insulin-like growth factor-1. Leptin can promote the initiation of sexual development and increase the secretion of sex hormones. There is a positive correlation between E_2_ and leptin, and there is also a positive correlation between leptin and FT3. Both E_2_ and FT3 can act on the ossification center of cartilage, which can increase the number of cells. Increased volume increases, accelerates the differentiation of cell morphology, advances bone maturation, and ultimately leads to accelerated bone age [17–19]. ② Excessive adipose tissue will produce more aromatase, which can induce androgen to be converted into estrogen. A high concentration of estrogen can promote the maturation and apoptosis of growth plate chondrocytes, and chondrocytes in the depleted hyperplasia layer can induce the fusion of the growth plate, which will accelerate the development of children's bone age. The secretion disorders of estrogen, testosterone, and insulin in overweight and obese children are all related to bone maturation, which adversely affects the speed of bone development [20, 21]. ③ Children and adolescents with excessive BMI usually have higher levels of adrenal androgen, thus increasing the secretion of leptin and increasing the risk of premature bone age [22].

Sexual development may be related to genetic susceptibility, diet, exercise, nutritional status, social economy, etc. Research by Liu et al. showed that the prevalence of precocious puberty after Tanner stage adjustment is 11.47% for girls and 3.26% for boys, and the incidence of precocious puberty in the obesity group is higher than that in the normal weight group [23]. Reinehr et al. investigated 160 overweight children and found that obese girls had earlier puberty, while obese boys showed delayed puberty [24]. In this study, there was a significant difference in the sexual development of children and adolescents under different nutritional status. Whether it was male or female, the sexual development of overweight and obesity was higher than that of the normal weight group in the same age group. Meanwhile, among female children, the sexual precocious puberty rate of the overweight + obesity group is higher. It is suggested that the sexual development of children and adolescents is closely related to their nutritional status. Some scholars believe that body fat can be transformed into estrogen. Compared with the normal population, obese girls are more likely to develop precocious puberty [25]. In addition, clinically, it is generally believed that overweight and obese people have high leptin levels, and leptin acts on the hypothalamus-pituitary-gonad axis, which can provide fat storage, promote the secretion of hypothalamic gonadotropin-releasing hormone, and increase the pulse frequency of luteinizing hormone, thus causing precocious puberty [26].

## 5. Conclusion

To sum up, the nutritional status of children and adolescents is closely related to their bone age and sexual development. People should pay more attention to the nutritional intake of children and adolescents, correct their partial and picky eating behaviors as early as possible, adjust the dietary structure, and increase food diversity. Parents also need to take reasonable measures to control the weight of children and adolescents, for example, ensuring regular meals, not overeating, choosing snacks reasonably, and actively carrying out physical activities. In addition, schools, communities, and medical and health institutions should work together to popularize nutrition and health knowledge among children, adolescents, and their parents, so as to ensure the balanced nutrition and physical health of children and adolescents. This study cannot dynamically observe the longitudinal development of bone age and sexual characteristics in children and adolescents, and it still needs to be further improved in future research.

## Figures and Tables

**Figure 1:** Relationship between nutritional status and early maturity of female children.

**Table 1:** Age distribution of 895 children and adolescents (*n*, %).

Age	Male (*n* = 466)	Female (*n* = 429)	Total (*n* = 895)
4 years∼	61 (13.1%)	28 (6.5%)	89 (9.9%)
6 years∼	82 (17.6%)	94 (21.9%)	176 (19.7%)
8 years∼	87 (18.7%)	192 (44.8%)	279 (31.2%)
10 years∼	150 (32.2%)	98 (22.8%)	248 (27.7%)
12 years∼	76 (16.3%)	17 (4.0%)	93 (10.4%)
14 years∼	10 (2.1%)	0 (0.0%)	10 (1.1%)

**Table 2:** Nutritional status and bone age level of children and adolescents (*n*, *M* ± SD).

Male	Age (years)	Bone age (years)	BAD	*F*_BAD_ value	*P*_BAD_ value
Emaciation group (*n* = 9)	9.10 ± 2.31	8.61 ± 2.39	−0.48 ± 1.39	20.38	<0.001
Normal group (*n* = 316)	9.25 ± 2.77	9.13 ± 3.15	−0.13 ± 1.08		
Overweight group (*n* = 88)	10.45 ± 2.21	10.88 ± 2.70	0.43 ± 1.12^#^		
Obesity group (*n* = 53)	9.52 ± 2.32	10.55 ± 2.83	1.03 ± 1.13^*∗*^^#△^		

Female	Age (years)	Bone age (years)	BAD	*F *_BAD_ value	*P*_BAD_ value
Emaciation group (*n* = 4)	9.15 ± 2.22	8.48 ± 1.84	−0.67 ± 1.08	20.33	<0.001
Normal group (*n* = 331)	8.98 ± 1.82	9.00 ± 2.35	0.01 ± 1.12		
Overweight group (*n* = 65)	8.76 ± 1.72	9.56 ± 1.88	0.80 ± 0.93^#^		
Obesity group (*n* = 29)	8.14 ± 1.77	9.42 ± 2.28	1.27 ± 0.87^*∗*^^#^		

*Note.* Compared with the emaciation group, ^*∗*^*P* < 0.05; compared with the normal group, ^#^*P* < 0.05; compared with the overweight group, ^△^*P* < 0.05.

**Table 3:** Nutritional status and bone age assessment of children and adolescents (*n*, %).

Male	Retardation of bone age	Normal bone age	Advancement of bone age	*χ* ^2^ value	*P* value	OR (95% CI)^*∗*^	OR (95% CI)^#^
Emaciation group (*n* = 9)	4 (44.44%)	4 (44.44%)	1 (11.11%)	63.55	<0.001	0.888 (0.108–7.292)	3.150 (0.822–12.067)
Normal group (*n* = 316)	64 (20.25%)	213 (67.41%)	39 (12.34%)			1.000	1.000
Overweight group (*n* = 88)	6 (6.82%)	52 (59.09%)	30 (34.09%)			3.674 (2.112–6.391)	0.288 (0.120–0.690)
Obesity group (*n* = 53)	2 (3.77%)	24 (45.28%)	27 (50.94%)			7.376 (3.911–13.909)	0.154 (0.037–0.651)

Female	Retardation of bone age	Normal bone age	Advancement of bone age	*χ* ^2^ value	*P* value	OR (95% CI)^*∗*^	OR (95% CI)^#^

Emaciation group (*n* = 4)	2 (50.00%)	2 (50.00%)	0 (0.00%)	71.11	<0.001	—	4.092 (0.566–29.599)
Normal group (*n* = 331)	65 (19.64%)	201 (60.72%)	65 (19.64%)			1.000	1.000
Overweight group (*n* = 65)	0 (0.00%)	38 (58.46%)	27 (41.54%)			2.908 (1.656–5.105)	—
Obesity group (*n* = 29)	0 (0.00%)	6 (20.69%)	23 (79.31%)			15.687 (6.137–40.099)	—

*Note.* ^*∗*^Compared with the normal group, the risk of advancement of bone age; ^#^compared with the normal group, the risk of retardation of bone age.

**Table 4:** Nutritional status and sexual development of children and adolescents (*n*, %).

Gender	Age	Normal group (developed/undeveloped, development rate)	Overweight + obesity group (developed/undeveloped, development rate)	OR (95% CI)
Male	6 years∼8 years	0/54 (0.00%)	0/24 (0.00%)	—
	8 years∼10 years	0/60 (0.00%)	3/26 (11.54%)	—
	10 years∼12 years	43/95 (45.26%)	30/52 (57.69%)	1.275 (0.717–2.267)

Female	6 years∼8 years	12/69 (17.39%)	9/24 (37.5%)	2.156 (0.808–5.752)
	8 years∼10 years	108/147 (73.47%)	36/44 (81.82%)	1.114 (0.672–1.847)
	10 years∼12 years	73/80 (91.25%)	15/16 (93.75%)	1.027 (0.474–2.225)

## Data Availability

All data included in this study are available upon request by contact with the corresponding author.
